This article has been retracted.

# Value of Humanized Nursing under Emergency Green Channel on Gastrointestinal Function Recovery in Patients with Acute Intestinal Obstruction after Operation

**DOI:** 10.1155/2023/2303766

**Published:** 2023-02-03

**Authors:** Siqi Luo, Yan Wang

**Affiliations:** The Nanhua Affiliated Hospital, Department of Operating Room, Hengyang Medical School, University of South China, Hengyang, Hunan 421001, China

## Abstract

Acute intestinal obstruction (AIO) is one of the most common surgical acute abdomens. Emergency green channel refers to a fast and efficient service system provided by hospitals for critically ill patients. It is the key to ensure that emergency patients receive timely, standardized, efficient and thoughtful medical services, improve the success rate of rescue, and reduce medical risks. Acute intestinal obstruction is mainly treated by surgery in the clinic. Previous reports have shown that the application of different nursing methods in the operation of acute intestinal obstruction has different effects on the results of surgical treatment. In this study, the clinical data of 80 patients with AIO were retrospectively analyzed to explore the value of humanistic care under the emergency green channel in promoting the recovery of gastrointestinal function after AIO surgery.

## 1. Introduction

Intestinal obstruction is an obstacle to the passage of intestinal contents caused by various reasons, which leads to clinical symptoms such as abdominal pain, constipation, vomiting, absence of defecation, and exhaustion in patients, and even results in systemic physiological disorders and endangers life safety [1]. Acute intestinal obstruction (AIO) is an extremely common type of intestinal obstruction, which has the characteristics of rapid onset, complex signs, and changeable causes [2]. Previous data revealed that AIO patients are unable to eat due to frequent vomiting, which can rapidly lead to decreased blood volume and hemoconcentration, and even endanger the life of patients when it is serious [3]. Therefore, surgical relief of intestinal obstruction remains the most immediate treatment option for AIO at this time.

Emergency green channel is a fast and efficient service system provided by hospitals for critically ill patients, which can ensure that standardized treatment can be convenient, efficient, and smooth and reach the hands of the crowd in urgent need of treatment. It has been verified in long-term practice that the application of emergency green channel greatly increases the rescue time of patients, prolongs their life cycle, and improves their prognosis and quality of life [4]. Based on this view, previous studies suggested that targeted psychological intervention combined with planned pain care could improve pain after AIO surgery [5]. Some studies also indicate that rapid rehabilitation nursing can promote postoperative recovery [6]. Previous literature studies have shown that humanized nursing can effectively reduce the perioperative adverse reactions of AIO patients and has application value [7]. This indicates that targeted care plays an extremely important role in improving surgical outcomes. Based on the above research, we believe that the humanized nursing under the emergency green channel has a significant effect on the recovery of gastrointestinal function of patients with AIO after surgery. Thus, this research will provide reliable theoretical guidance for future clinical treatment by analyzing the effectiveness of humanized nursing.

## 2. Materials and Methods

### 2.1. General Information

80 patients with AIO admitted to the emergency department of our hospital from January 2020 to December 2021 were selected for the retrospective analysis. Among them, 37 patients who received the conventional nursing intervention under the emergency green channel were regarded as the control group, while 43 with the humanized nursing intervention were enrolled in the research group.

### 2.2. Inclusion and Exclusion Criteria

Inclusion criteria were as follows: age >18, confirmed as AIO by clinical tests and imaging examinations, and the symptoms were fully consistent with the signs of AIO onset [8]; patients who met the surgical indications [9]; complete medical records; those agreed to participate in this research. Exclusion criteria were as follows: those with abnormal heart, liver, and kidney functions; those with mental abnormalities and communication disorders; those with contraindications to surgery or medications; patients transferred to other hospitals; those with low treatment compliance.

## 3. Methods

### 3.1. Establishment of Emergency Green Channel

All departments of the hospital had standardized the diagnosis and treatment procedures of the green channel and set up special emergency telephone numbers for the green channel. After a patient visited a doctor, the doctor visiting the doctor must quickly clarify the condition and determine the main factors affecting the life of the patient. Rescue orders, consultation orders, inspection orders, and surgical orders are issued. Emergency drugs, especially shock drugs, in time according to the patient's condition are prepared. Meanwhile, appropriate doctors should be contacted in advance for further treatment, and the operating room should be informed timely to prepare for the corresponding surgery. At the same time, emergency department nurses quickly created venous access, instructed him to remain supine, completed oxygen dosing, and created cardiac monitoring. And a blood sample is collected for standby. In the process of emergency treatment, we should closely observe the changes in his condition to ensure the smooth flow of fluid and blood and assist doctors in handling it.

### 3.2. Nursing Methods

#### 3.2.1. Control Group

Patients received routine nursing interventions after being transferred to the department from the emergency room. Nursing staff first registered patients' physical conditions, then conducted health education, instructed them on how to regulate their diet, monitored their vital signs in real time, made preoperative preparations, helped them to carry out surgical treatment smoothly, and implemented routine anti-infection measures after surgery until they were discharged from the hospital.

#### 3.2.2. Research Group

Patients received humanized nursing after being transferred from the emergency department to the department for treatment. ① A personalized nursing group headed by the head nurse of the department is established in the department. All team members receive relevant training. ② Understand the actual needs, pain, psychology, diet, adaptation, and other conditions of each patient, and give corresponding preoperative care. At the same time, the patients were educated about the disease and the previous successful cases, so that they could understand the disease, reduce anxiety, and improve compliance. Besides, the operating procedures were carefully explained, and precautions were informed in advance to make patients feel relaxed. Strictly observe the changes in vital signs to promote the optimal implementation of the surgery. ② The patients were guided to be in the semilying position after the anesthesia disappeared, in order to promote the recovery of intestinal function, and timely intervention was given to severe pain. ③ After the operation, we formulated a diet plan for the patient and tried to take liquid food in the initial stage of treatment to minimize the stimulation to the digestive tract. On an empty stomach, small amounts of liquid, semiliquid, and coarse fiber foods are used as directed by your doctor to promote airflow. Patients are regularly assisted in expectoration, turning over, and the like, and are encouraged to perform the functional exercise as soon as possible and to get out of bed after the condition is stable. Instruct them to proceed gradually until discharge.

### 3.3. Observation Index

1. Postoperative recovery: The time of first anal discharge, first bed activity, intestinal function recovery, and the length of stay after surgery were counted in both groups.
2. Nursing efficacy: Cured: The clinical symptoms such as nausea, vomiting, and abdominal pain completely disappeared. Patients could defecate and ventilate, and they could eat semiliquid food. Improved: The clinical symptoms are relieved, and patients can defecate, pass gas, and consume semiliquid food. Ineffective: No change or worsening of clinical symptoms. Total effective rate of nursing = (cured + improved)/total × 100%.
3. Pain: Patients' pain before and after nursing was assessed via the visual analogue scale (VAS) and the general comfort questionnaire scale (GCQ), with the VAS scoring out of 10 and higher scores representing more marked pain; the full score of GCQ is 80, and the higher the score, the higher the comfort.
4. Psychology: The psychology of patients before and after nursing was evaluated via anxiety rating scale (SAS) and depression rating scale (SDS). The decrease in score indicated the decrease in negative emotions, such as anxiety and depression.
5. Adverse reactions: Patients were counted for adverse reactions that occurred between the postoperative period and discharge, and the incidence rate was calculated.
6. Quality of life: The quality of life of patients after nursing was assessed via the generic quality of life inventory-74 scale (GQOL-74), and the scores included mental function, physical function, material life, and social function, with higher scores indicating higher quality of life.
7. Nursing satisfaction: Patients were discharged from the hospital with a nursing satisfaction survey, which was divided into four levels: very satisfied, satisfied, needs improvement, and unsatisfied.

### 3.4. Statistical Methods

Data were statistically analyzed via SPSS 23.0 software. Measurement data were expressed as mean ± standard deviation ($\bar{x}$ ±*s*), independent sample *t*-test was used for comparison between groups, count data were expressed as [*n*(%)], and chi-square (*χ*^2^) test was performed. The differences were statistically obvious (*P* < 0.05).

## 4. Results

### 4.1. Comparison of Clinical Baseline Data between the Two Groups

There were no statistically marked differences in terms of age, gender, type of AIO, BMI, nationality, family history of disease, history of smoking, and history of drinking (*P* > 0.05), indicating comparability between groups (Table 1).

### 4.2. Comparison of Postoperative Recovery between the Two Groups

The time of first anal discharge, first bed activity and intestinal function recovery, and the length of hospital stay after surgery were shorter in the research group than in the control group (*P* < 0.05, Figure 1).

### 4.3. Comparison of Nursing Efficiency before and after Nursing between the Two Groups

The total nursing efficiency of the research group was 88.37%, and the difference was statistically dramatic compared with that of the control group of 70.27% (*P* < 0.05, Table 2).

### 4.4. Changes of Pain before and after Nursing between the Two Groups

There was no significant difference in VAS and GCQ scores before nursing (*P* > 0.05). After nursing, the VAS score of patients in the two groups was decreased and was lower in the research group than in the control group; the GCQ score of the two groups was increased and was higher in the research group than in the control group (*P* < 0.05, Figure 2).

### 4.5. Changes in Psychology before and after Nursing between the Two Groups

There was no difference in SAS and SDS scores between groups before nursing (*P* > 0.05), and both decreased after nursing, and the research group was lower than the control group (*P* < 0.05, Figure 3).

### 4.6. Comparison of Adverse Reactions between the Two Groups

The incidence of adverse reactions in the research group was 9.30%, which was lower than that in the control group (27.03%) (*P* < 0.05, Table 3).

### 4.7. Comparison of Quality of Life between the Two Groups

The GQOL-74 scores in both groups denoted that the four dimensions of somatic function, psychological function, social function, and material function were higher in the research group than in the control group (*P* < 0.05, Figure 4).

### 4.8. Comparison of Nursing Satisfaction before and after Nursing between the Two Groups

There was no marked difference in the number of nursing satisfaction such as satisfied, needing improvement, and unsatisfied (*P* > 0.05), but that of very satisfied was 55.81% in the research group, which was higher than the control group (29.73%) (*P* < 0.05) (Table 4).

## 5. Discussion

AIO, as an extremely common intestinal disorder, will potentially endanger patients' lives if not treated promptly and appropriately [10]. Currently, the number of new cases of AIO worldwide is increasing year by year. How to effectively, quickly, and accurately save the life of a patient has become a hot topic in clinical research.

The traditional emergency admission process is complicated and can easily delay the “golden time” of emergency care [11, 12]. As the latest concept proposed in emergency departments, the emergency green channel has been proven to be excellent in the success rate of rescuing patients with acute diseases such as ischemic stroke and amputation, and it is equally applicable to AIOs that require rapid surgical management [13, 14]. At present, emergency green channels have been more and more frequently used clinically [15, 16]. The emergency green channel allows for a clear distribution of work among the various departments in the emergency process and facilitates the smooth operation of emergency care. In addition, the emergency green channel is also conducive to improving the emergency rescue ability of nursing staff, prompting them to continuously improve their business level and nursing skills, so that they can handle complex injuries without fear, cooperate with anesthesiologists and surgeons to complete surgery in an orderly manner, and improve the success rate of surgical rescue for traumatic shock patients [17]. Opening an emergency green channel can also prioritize the implementation of relevant examinations, laboratory tests, treatments, and surgeries, ensuring that the relevant departments can complete the diagnostic and treatment examinations in the shortest possible time, thus shortening the preparation time for emergency treatment [18, 19]. This not only can greatly protect the life safety of AIO patients but also facilitate better clinical control of their pathological changes, thus enhancing their postoperative recovery to a certain extent. Zhang et al. confirmed that the postoperative recovery time of AIO patients was longer than that of patients in the current study [11], which was also related to the implementation of the emergency green channel. AIO is a high-risk disease with rapid progression and may pose a high risk of death if not rescued in time.

However, it is known that patients with AIO usually need to stay in bed for a long time after surgery. In this process, nursing staff should pay attention to provide targeted care from the perspectives of vital signs, gastrointestinal conditions, complications, and mentality and assist clinicians in giving appropriate treatment and dietary medication guidance [12]. In this study, the recovery conditions of patients after surgery were first compared. The patients in the research group had a shorter time to exhaust gas for the first time, time to get out of bed, and time to recover intestinal function and hospital stay after surgery than those in the control group. The total effective rate of the former was higher than that of the latter, which fully illustrated the high recovery efficiency of patients in the research group. Second, through the comparison of patients' pain, it was found that the VAS score of the research group was lower than that of the control group, while the GCQ score was higher, indicating that the pain in the research group after surgery was lower. Humanistic care under the emergency green channel can improve patients' postoperative pain and recovery. In previous studies, we also found that humanized nursing could shorten the postoperative rehabilitation process of patients with tumor combined with mental disorders [20, 21], which could also verify the accuracy of the results of the experiment. Therefore, we believe that humanistic care in the green channel of emergency room can effectively improve the therapeutic effect of AIO and provide more reliable safety guarantee for patients. To analyze the reasons, in conventional nursing care, nursing staff cannot meet the expected satisfaction for all these aspects, so there may be some limitations in the patient's postoperative rehabilitation. Humanistic care is a targeted nursing strategy targeted at the psychological and physiological levels of patients, which is more easily accepted by patients due to their individual differences. In humanized nursing, nursing staff should pay attention to patients' own feelings, plan diet and rehabilitation according to patients' condition, patiently explain the importance and scheme of treatment, and answer all questions raised by patients, so that they can have a deeper understanding of the development of the disease and effectively alleviate their negative psychology and emotions [22].

In this study, the SAS and SDS scores of the two groups were further compared, and the results showed that the improvement degree of SAS and SDS in the research group after the intervention was more significant than that in the control group. This finding was consistent with that of Zeng and Guan [23], and it could reaffirm the application value of humanized nursing. The reason was that humanistic nursing intervention could not only transmit disease-related knowledge to patients through a variety of ways under the basic premise of conventional drug treatment, strengthen their understanding and mastery of disease factors, clinical manifestations, precautions, and other related content, and then improve the patients' bad psychology. In addition, targeted care can also promote them to form a good lifestyle and habits, and reduce the recurrence of diseases caused by poor living habits. Therefore, the incidence of postoperative adverse reactions in the study group was lower than that in the control group. The improvement in quality of life throughout the nursing service naturally enhances the subjective feelings of the patient. Therefore, the quality of life in the research group after surgery was superior to that in the control group, and the degree of nursing satisfaction was high, which fully illustrated the applicability of humanized nursing in AIO.

In conclusion, humanized nursing under the emergency green channel can effectively enhance the recovery and comfort of postoperative gastrointestinal function and reduce adverse effects in AIO patients, thus having high clinical application value. Nevertheless, due to the short experimental period, we are unable to evaluate the long-term prognosis of both groups, which is still worthy of future follow-up investigation. Besides, we need to increase the number of cases studied to obtain more comprehensive results for clinical reference.

## Figures and Tables

**Figure 1:** Postoperative recovery between two groups. Note: (a) comparison of time of first anal discharge; (b) comparison of time of first bed activity; (c) comparison of time of intestinal function recovery; (d) comparison of length of hospital stay. ^*∗*^*P* < 0.05.

**Figure 2:** Comparison of pain between two groups. Note: (a) comparison of VAS scores before and after nursing; (b) comparison of GCQ scores before and after nursing. ^*∗*^*P* < 0.05.

**Figure 3:** Comparison of changes in psychology between two groups. Note: (a) comparison of SAS scores before and after nursing; (b) comparison of SDS scores before and after nursing. ^*∗*^*P* < 0.05.

**Figure 4:** Comparison of GQOL-74 scores. Note: (a) comparison of somatic function scores; (b) comparison of psychological function scores; (c) comparison of social function scores; (d) comparison of material function scores. ^*∗*^*P* < 0.05.

**Table 1:** Comparison of clinical baseline data.

	Control group (*n* = 37)	Research group (*n* = 43)	*t*/*χ*^2^	*P*
Age	54.32 ± 4.06	55.72 ± 4.72	1.410	0.163
Gender			0.131	0.717
Male	28 (75.68)	34 (79.07)		
Female	9 (24.32)	9 (20.93)		
Type of AIO			0.754	0.860
Dynamic intestinal obstruction	8 (21.62)	8 (18.60)		
Hematogenous intestinal obstruction	9 (24.32)	11 (25.58)		
Incomplete intestinal obstruction	14 (37.84)	14 (32.56)		
Strangulated intestinal obstruction	6 (16.22)	10 (23.26)		
BMI (kg/m^2^)	26.62 ± 2.84	26.13 ± 2.38	0.840	0.404
Nationality			0.037	0.848
Han nationality	34 (91.89)	40 (93.02)		
Ethnic minorities	3 (8.11)	3 (6.98)		
Family history of disease			0.119	0.730
Yes	5 (13.51)	7 (16.28)		
No	32 (86.49)	36 (83.72)		
Smoking			0.224	0.636
Yes	30 (81.08)	33 (76.74)		
No	7 (18.92)	10 (23.26)		
Drinking			0.159	0.690
Yes	19 (51.35)	24 (55.81)		
No	18 (48.65)	19 (44.19)		

**Table 2:** Comparison of nursing efficiency.

Group	Cured	Improved	Invalid	Total effective rate (%)
Control group (*n* = 37)	12 (32.43)	14 (37.84)	11 (29.73)	70.27
Research group (*n* = 43)	24 (55.81)	14 (32.56)	5 (11.63)	88.37
*χ * ^2^				4.073
*P*				0.044

**Table 3:** Comparison of adverse reactions.

Group	Incision cracking	Intraperitoneal infection	Anastomotic fistula	Gastrointestinal dysfunction	Incidence of adverse reactions (%)
Control group (*n* = 37)	2 (5.41)	1 (2.70)	3 (8.11)	4 (10.81)	27.03
Research group (*n* = 43)	1 (2.33)	0 (0.00)	1 (2.33)	2 (4.65)	9.30
*χ * ^2^					4.328
*P*					0.038

**Table 4:** Comparison of nursing satisfaction.

Group	Very satisfied	Satisfied	Needing improvement	Unsatisfied
Control group (*n* = 37)	11 (29.73)	14 (37.84)	8 (21.62)	4 (10.81)
Research group (*n* = 43)	24 (55.81)	12 (27.91)	5 (11.63)	2 (4.65)
*χ * ^2^	5.498	0.894	1.459	1.088
*P*	0.019	0.344	0.227	0.297

## Data Availability

The data can be obtained from the author upon reasonable request.
